# Adolescent Mental Health Literacy Questionnaire: Investigating Psychometric Properties in Iranian Female Students

**DOI:** 10.1155/2022/7210221

**Published:** 2022-05-18

**Authors:** Somayeh Zare, Mohammad Hossein Kaveh, Ahmad Ghanizadeh, Mahin Nazari, Abdolrahim Asadollahi, Razie Zare

**Affiliations:** ^1^Department of Health Promotion, School of Health, Shiraz University of Medical Sciences, Shiraz, Iran; ^2^Department of Psychiatry, School of Medicine, Shiraz University of Medical Sciences, Shiraz, Iran; ^3^Department of Industrial & Organizational Psychology, Faculty Education & Psychology, Shahid Chamran University, Ahvaz, Iran

## Abstract

**Objectives:**

Mental Health Literacy (MHL) is an important factor in promoting mental health. Assessing this structure is required for early recognition and intervention in mental health problems. To date, there was no tool to assess it among Iranian adolescents, so this study was aimed at examining the psychometric properties of the Persian version of the Adolescent Mental Health Literacy Questionnaire (AMHLQ) among Iranian female students.

**Method:**

The study instrument was a Persian version of the AMHLQ prepared through a translation and back-translation process. In this cross-sectional study, 275 female students completed the AMHLQ, and the Adolescent Strengths, and Difficulties Questionnaire (SDQ).

**Results:**

Findings of content, construct validity tests, Cronbach's alpha, and split-half coefficient demonstrated that the AMHLQ had satisfactory validity and suitable reliability. The exploratory factor analysis showed four dimensions of the AMHLQ: (1) knowledge of mental health problems (*α* = 0.89); (2) erroneous beliefs/stereotypes (*α* = 0.89); (3) help-seeking and first aid skills (*α* = 0.86); and (4) self-help strategies (*α* = 0.74).

**Conclusion:**

The findings showed that the tool was confirmed by questions and subscales, and this questionnaire was a valid and reliable tool in assessing level differences of MHL and in determining the impact of programs designed to improve MHL in Iranian female adolescents.

## 1. Introduction

Mental health problems are one of the leading causes of illness in the world [1]. Adolescence is a critical period for mental health disorders. Research has shown that the prevalence of adolescent mental health problems in different countries is increasing [2]. For many people, the symptoms of mental illness first appear before the age of 14 [3]. It is estimated that mental health disorders affect approximately 13.4% of children and adolescents worldwide, and this poses a significant threat to the health and well-being of young people [4]. About one-fifth of children and adolescents in Iran suffer from at least one mental disorder [5]. The prevalence of mental health problems in adolescents in southern Iran was 22.38%, in Kurdistan 33.8%, in Semnan 24.8%, and in Tehran 28.2% [6–9]. The prevalence of mental health disorders is higher in girls than in boys [10, 11]. The prevalence of major depression in female students was 52.6% in the city of Hamadan, in western Iran [12].

Mental problems during adolescence can lead to long-term dysfunction in adulthood [13]. The impact of these problems on students' learning and overall functioning is undeniable. Students with mental health problems achieve low academic achievement. They are less involved in school, have poor relationships with their peers and parents, and are more likely to drop out [14, 15].

Despite the high prevalence of mental health disorders, there is a significant treatment gap between requesting and receiving care. One of the main reasons for this gap is the low level of Mental Health Literacy (MHL) [16]. Various studies have shown that MHL is a good determinant of mental health in adolescents [17, 18]. The term MHL was first used by Jorm et al. (1997) to refer to knowledge and beliefs about mental disorders that help to recognize, manage, or prevent them. MHL includes the ability to recognize specific disorders, knowledge of how to seek mental health information, knowledge about risk factors and causes, self-treatments, and professional help available, and attitudes that promote recognition and appropriate help-seeking [19, 20]. Understanding the nature and effect of MHL has shifted from its primary focus as information about mental disorders to a more comprehensive structure called empowerment competency [19, 21]. The recent definition of MHL includes four distinct components: understanding how to achieve and maintain good mental health, understanding mental disorders and their treatment, reducing stigma, and increasing the effectiveness of help-seeking (knowing when and where evidence-based mental health care can obtain and having the competence to increase self-care) [21, 22]. Studies have shown that young people have similar MHL deficiencies as adults [19, 23, 24]. A review study investigating the health literacy status of adolescents stated that 83.6% of students had an inadequate MHL level [25].

In general, young people have little positive attitude about professional help (meeting with a psychologist or psychiatrist). Many young people prefer to talk to a family member when they have a mental health problem [26]. MHL is recognized as a prerequisite for early recognition and intervention in mental disorders [27]. Evidence suggests that people with adequate MHL can detect early-stage mental health disorders, are more likely to seek professional help, and have fewer stigmatizing attitudes [28]. By assessing one's knowledge and beliefs, we can identify the stigma that is related to one's mental health problems, which is one of the main barriers to early recognition and intervention [29]. People with higher MHL are likely to be better able to recognize mental illness and identify appropriate treatment resources, while lower MHL is associated with early termination of mental health treatment and the use of inappropriate coping strategies such as using alcohol and other medications [30].

The assessment of MHL enables the development of interventions aimed at promoting MHL as well as the evaluation of these interventions [31]. Also measuring MHL at a community level is critical to promoting mental health care [30]. Several studies have developed and reviewed the psychometric properties of the questionnaire to measure MHL. Bjørnsen et al. developed the MHPK-10 questionnaire as a measure of mental health promotion with ten items and one factor for measuring the knowledge of factors affecting mental health in adolescents [32]. Castellvi Obiols et al. prepared and validated the http://EspaiJove.net MHL (EMHL) questionnaire to assess the MHL of Spanish adolescents in a sample of 13-15 years old students (355 people). The final version of that questionnaire had 35 items and two sections. The first part is a dual choice format (yes/no) to identify mental disorders, and the second part is a multiple-choice question with four possible answer options [33]. Chao et al. has developed a MHL questionnaire for healthcare students. It has 26 items and five factors for maintaining positive mental health, diagnosing mental illness, attitudes about the stigma of mental illness, the effectiveness of help-seeking, and attitudes about help-seeking [34]. These tools had some limitations were included: assessing only one dimension of MHL, such as the dimension of knowledge, having lower psychometric properties, and using multiple-choice questions, administering to older than 17 years, and the special population such as medical and public health students. A review study showed that although the studies used different methods in adolescent MHL interventions, they all had a positive effect on MHL levels, and given that self-report assessment was used to measure MHL in these studies, confirmation of these results is still needed using objective tools [35].

Therefore, there is a need for a suitable tool to evaluate the level of MHL in adolescents. Due to the lack of an instrument to measure MHL among Iranian adolescents, this study was conducted to examine the psychometric properties of the Persian version of the MHL questionnaire developed by Campos et al. [29] among Iranian female adolescents.

## 2. Methods

This cross-sectional study was conducted to evaluate the validity and reliability of the AMHLQ among Iranian female students.

### 2.1. Participants

To estimate sample size was based on the recommendation of having five to ten participants per the scale's items [36, 37]. Participants in the study included 275 female students in the eighth grade with a mean age of 13.80 and a standard deviation of 0.66. They were studying in public schools in Shiraz. Permissions were achieved from the Shiraz University of Medical Science and the Ministry of Education, Shiraz, and from the school administrators for collecting survey data from students. The cluster random sampling method was conducted among Shiraz's four education districts. From the four districts, two districts were selected randomly (districts 1 and 3). In each of the selected districts, four public schools were randomly selected. In each school, two classes were randomly selected, and eventually, 275 female students were selected. The inclusion criteria were as follows: studying in Shiraz public schools, studying in the eighth grade, agreeing to participate in the study, and filling out an informed consent form.

### 2.2. Measures

Data collection tools include the Adolescent Mental Health Literacy Questionnaire (AMHLQ) and the Persian version of the Adolescent Strengths and Difficulties Questionnaire (SDQ).

#### 2.2.1. Adolescent Mental Health Literacy Questionnaire

This questionnaire was developed by Campos, and it contains 33 items on a Likert scale (from 1 = strongly disagree to 5 = strongly agree), which is organized in three dimensions: [1] knowledge/stereotypes (18 items); [2] first aid skills and help-seeking (10 items); and [3] self-help strategies (5 items). The questionnaire assesses the following: [1] knowledge of mental health issues, including general characteristics of mental health problems, prevalence, signs, and symptoms, and risk factors for mental disorders, as well as protective factors/mental health promoters; [2] knowledge of three specific mental disorders—depression, anxiety, and eating disorders; [3] stereotypes associated with mental disorders; and [4] behavioral intentions (predisposition to help, mental health behavioral promoters, self-help strategies, and behaviors that promote formal and/or informal seeking help). In the main study, the questionnaire showed good internal consistency (*α* = 0.84) [29]. The original version is about three disorders: depression, anxiety, and schizophrenia, but the researchers based on an interview with a panel of experts as well as a review of previous studies that have shown that the prevalence of eating disorders is high in girls replaced two schizophrenic questions with two questions about eating disorders [38–43]. So item 4 was replaced with this item: Anorexia nervosa is a type of eating disorder that can lead to death. Item 31 was replaced with this item: In bulimia nervosa, to compensate for the overeating and to prevent weight gain, the person is forced to vomit or to exercise vigorously, or using laxatives inappropriately.

#### 2.2.2. Strengths and Difficulties Questionnaire (SDQ)

This questionnaire was developed by Goodman in the UK (1997) and is used for ages 4 to 16 [44, 45]. It has 25 items and five subscales of hyperactivity scale, emotional symptom scale, conduct problem scale, peer problem scale, and prosocial scale (child strengths). Measurements of the answers in the questionnaire are based on a 3-point Likert scale (“not true,” “somewhat true,” or “certainly true”). We used the Persian version of the SDQ. The study of Ghanizadeh and Izadpanah supports the good psychometric properties of the Persian version of the SDQ [46].

### 2.3. Translation of AMHLQ

The translation of the AMHLQ from English to Persian was conducted based on World Health Organization guidelines in four sequential steps [47]. In translating this questionnaire, an attempt was made to translate vocabularies, idioms, and interpretations nonliterally, and technical words and terms were avoided as much as possible [48]. Linguistic structures were also used that could be understood by Persian speakers. First, two bilingual native Iranians (Persian-English) with knowledge of psychology and health professional translated the questionnaire from English to Persian. Second, in the experts' panel, they discussed the translated version until reaching a consensus. For example, in item 19, “to go to a doctor” was replaced “to get medical support.” Third, the original forward Persian translation was back-translated by an independent English-language translator, a native English speaker who was not aware of the original English version. Fourth, the translations were reviewed by a panel of experts. No significant differences were identified between the Persian version of the MHL measure and the original version of the MHL measure.

### 2.4. Ethics Considerations

All participants signed informed consent forms. The ethics committee has approved this study at Shiraz University of Medical Sciences. The ethical code is IR.SUMS.REC.1398.676.

### 2.5. Data Analysis

To analyze the collected data, SPSS-26 and AMOS-24 software were used. Two methods of qualitative and quantitative content validity were used to evaluate the content validity index. In the qualitative content validity method, the tool was given to 15 specialists in the field of health education, psychologist, and psychiatrist. They were asked to provide the necessary feedback after a qualitative review of the questionnaire based on the criteria of compliance with grammar, use of suitable words, placement of phrases in grammar, use of appropriate words, placement of phrases in their proper place, and appropriate scoring. These specialists were also consulted about the face validity of the questionnaire. The content validity index was used quantitatively to confirm the validity of the content. This indicator was used to assess the three criteria of simplicity and fluency, relevance and clarity, or transparency using the 4-point Likert spectrum as follows: **(**A) The criterion of simplicity and fluency: it is complex, it needs serious review, it is simple, but it needs to be reviewed, and it is quite simple. (B) The criterion of relevance: it is not related at all, it is somewhat related, it is relatively related, and it is completely related. (C) The criterion of clarity and transparency: it is vague, it needs serious review, it is clear, but it needs to be reviewed, and it is quite clear [49]. If the number of specialists in this section is 15, according to Lynn's guidelines [50], the items will remain in the questionnaire with a score of more than 0.79. If the score of the index is between 0.70 and 0.79, the phrase is questionable and needs to be corrected and revised. And if the index score is less than 0.70, the phrase is unacceptable and should be deleted [50]. The formula used for the content validity index at this stage was as follows: the number of people who scored 3 or 4 on the relevant question/the total number of scorers.

To evaluate construct validity, firstly, the construct validity of the AMHLQ was determined to extract the number of hidden factors using exploratory factor analysis. Secondly, to assess the fitness of the final model of the four-factor structure of AMHLQ, confirmatory factor analysis was performed. It should be noted before analyzing the data to ensure that the research data meets the underlying assumptions of confirmatory factor analysis such as missing data and to perform analysis on complete data without missing values was used from the missing data replaced with the mean method. For the assessment of the model fit, the value of the chi-square index, normed *χ*^2^ measure index (the chi-square ratio of the degree of freedom), Goodness of Fit Index (GFI), Adjusted Goodness of Fit Index (AGFI), Normed Fit Index (NFI), Comparative Fit Index (CFI), Incremental Fit Index (IFI), Tucker-Lewis Index (TLI), and Root Mean Squared Error of Approximation (RMSEA) were used. To obtain more evidence to validate the AMHLQ, the correlation of the dimensions of this scale with the SDQ was used to assess concurrent validity. Reliability was assessed by measuring internal consistency with Cronbach's alpha and split-half technique.

## 3. Results

### 3.1. Sample Characteristics

In the present study, 275 female students in the eighth grade participated. Among the participants, 5.5% (*n* = 15) reported a family history of mental illness, 53.81% (*n* = 148) had no family history of mental illness, and 40.72% (*n* = 112) did not answer. They reported that 7.6% of mothers (*n* = 21) were employee, 84.4% of them (*n* = 232) were housewife, 7.6% of them (*n* = 21) had free business, and 0.4% (*n* = 1) did not answer. 21.5% of father's occupation (*n* = 59) were employee, 12% (*n* = 33) were workers, 53.5% (*n* = 147) were self-employed, 4.7% (*n* = 13) were retired, 4.7% (*n* = 13) were unemployed, and 3.6% (*n* = 10) did not answer.

### 3.2. Content Validity

The results of content validity are presented in Table 1. All items have a score higher than 0.79. So all the items remained.

### 3.3. Construct Validity

#### 3.3.1. Exploratory Factor Analysis

For the questionnaire, assumptions for exploratory factor analysis were confirmed (Kaiser-Meyer-Olkin = .92, Bartlett's test of sphericity =5233.81, df = 528, *p* < .001). The results of these indicators show a good correlation between the variables that allow factor analysis. The factors hidden in the questionnaire were extracted by principal component analysis and varimax rotation. In this model, four factors were extracted according to eigenvalues higher than one. The four hidden factors after rotation had eigenvalues of 12.57, 2.86, 1.49, and 1.29, respectively. The four extracted factors explained 58.89% of the total variance of the construction of the AMHLQ in students. The exploratory factors extracted from the AMHLQ have been presented in Table 2.

#### 3.3.2. Confirmatory Factor Analysis

Confirmatory factor analysis was performed to assess the fitness of the final model of the four-factor structure of the MHL questionnaire. The factor structure of the AMHLQ in the present study has been presented in Figure 1.

Figure 1 shows that all items had moderate to high factor loads (*p* < 0.001). A value of 0.40 is the acceptable cut-off point in most cases for confirmatory factor analysis [51]. Additionally, the indicators of the confirmatory factor analysis model of AMHLQ demonstrated that the measures of the indicators were close to the fitness criteria and that the confirmatory factor analysis model had an acceptable fit [52]. The fitness indicators of the factor analysis model of AMHLQ have been presented in Table 3.

According to Table 3, the fitness indices of the confirmatory factor analysis model in the AMHLQ in the present study were acceptable.

### 3.4. Concurrent Validity

The descriptive indicators of AMHLQ and SDQ based on the central indicators and dispersion have been presented in Table 4, and the results related to validity have been presented in Table 5.

Regarding concurrent validity, the results of the Pearson correlation showed that there is a negative correlation significantly between the Persian version of the AMHLQ and the SDQ.

### 3.5. Reliability

To evaluate the reliability of AMHLQ, Cronbach's alpha and split-half methods were used, and the results of which have been reported in Table 6.

## 4. Discussion

The primary purpose of the study was to examine the psychometric properties of a Persian version of the AMHLQ in a sample of Iranian girl high-school students. The results of qualitative and quantitative content validity analysis showed that the translated AMHLQ has a satisfactory content validity and was appropriate for assessing MHL in Iranian girl high school students. Cronbach's alpha coefficient was used to determine internal consistency. The reliability coefficient of the whole questionnaire was 0.94, which indicated that the questionnaire had a coherent structure. These results were consistent with Dias et al.'s study. In this study, the questionnaire showed good internal consistency (*α* = 0.84) [31]. Also, the results of the reliability coefficient obtained using the split-half method were 0.87, which indicated the acceptable reliability of the Persian version of AMHLQ [53]. In the present study, the factor fitness of the AMHLQ was evaluated using confirmatory factor analysis, and the most common fitness indicators of the model were evaluated. The results of model fitness were evaluated as appropriate for all indicators, and all factor loads were above 0.4, which indicated that they had the minimum acceptable amount of factor load. The results of exploratory factor analysis showed four dimensions of AMHLQ that were consistent with the multidimensional perspective of the construct of MHL and the results of the Dias et al. study [31]. According to the results of exploratory factor analysis, one item (If I had a mental disorder I would seek friends' help) is in the erroneous beliefs/stereotypes dimension, while in the main questionnaire, it was in the first aid skills and help-seeking behavior dimension. This difference may be due to the cultural differences of the study participants. Culture could account for health-seeking behavior, type of services and support system, and variations in how people communicate their health concerns. Culture also influences the meanings that people impart to their illness and also the stigma associated with such illnesses [54]. The concurrent validity of the questionnaire also showed a significant negative correlation between the Persian version of adolescent MHL with the SDQ, which yielded similar results to Castellvi et al.'s research [33]. Adolescents who score lower on the dimensions of MHL have more behavioral and emotional problems.

## 5. Limitations and Implications

Our study has some limitations. The main limitation of the study is that it was performed only on eighth-grade girls in Shiraz, and this reduces the generalizability of the results in boys, of other ages, and other cultures. Despite this limitation, the present questionnaire focuses on the majority of aspects of MHL compared to many other tools. It is therefore a concise and cost-effective tool for examining knowledge about mental health problems, misconceptions/stereotypes, first aid skills and seeking help behaviors, and self-help strategies. Assessing the psychometric properties of this questionnaire is recommended for boys and other ages. Further research is recommended for the cross-cultural validation of this instrument.

## 6. Conclusion

The findings showed that the tool was confirmed by questions and subscales. This study provides initial support for the use of the AMHLQ among Iranian girl high-school students. The results showed that the translated AMHLQ is a suitable tool to assess MHL in girl adolescents that could be used by psychologists and counselors. This questionnaire is an efficient tool for educators and researchers to design and implement adolescent health promotion programs in research settings, planning mental health promotion activities, and evaluating public mental health education initiatives for students.

## Figures and Tables

**Figure 1:** Confirmatory factor analysis of AMHLQ.

**Table 1:** Validity index rate of AMHLQ items.

Specify your agreement on each of the following statements	Simplicity and fluency (1 to 4)	Related (1 to 4)	Clarity and transparency (1 to 4)
Item 1	1	1	1
Item 2	1	0.80	1
Item 3	0.80	0.93	0.93
Item 4	1	0.80	1
Item 5	0.93	0.80	0.93
Item 6	1	1	1
Item 7	0.93	0.80	1
Item 8	0.80	0.80	0.93
Item 9	1	0.93	1
Item 10	1	0.80	0.93
Item 11	1	0.80	0.93
Item 12	1	1	1
Item 13	0.80	0.80	0.93
Item 14	1	0.86	1
Item 15	1	0.80	1
Item 16	0.93	0.86	1
Item 17	1	0.80	1
Item 18	0.93	0.80	0.93
Item 19	1	0.80	1
Item 20	1	0.86	1
Item 21	1	0.93	1
Item 22	1	0.93	1
Item 23	0.80	0.93	0.80
Item 24	1	0.80	1
Item 25	1	0.80	1
Item 26	1	0.80	1
Item 27	1	1	1
Item 28	1	1	1
Item 29	1	0.93	1
Item 30	1	0.86	1
Item 31	0.80	0.80	0.93
Item 32	0.93	0.80	0.93
Item 33	1	0.93	1

**Table 2:** Exploratory factors extracted from the AMHLQ.

Factor	No	Items	Factor loadings	Items share	Eigenvalues
Erroneous beliefs/stereotypes	28	Depression is not a true mental disorder.	-0.727	0.639	12.57
	30	Only adults have mental disorders.	-0.696	0.608	
	29	Mental disorders do not affect people's behaviors.	-0.666	0.599	
	31	The sooner mental disorders are identified and treated, the better.	0.657	0.618	
	33	Mental disorders do not affect people's feelings.	-0.645	0.592	
	32	If a friend of mine developed a mental disorder, I would listen to her/him without judging or criticizing.	0.643	0.596	
	27	If a friend of mine developed a mental disorder, I would not be able to help her/him.	-0.613	0.591	
	25	People with mental disorders come from families with little money.	-0.583	0.533	
	23	If I had a mental disorder, I would seek my friends' help.	0.561	0.583	
Knowledge of mental health problems	6	Mental disorders affect people's thoughts.	0.801	0.713	2.86
	5	Drug addiction may cause mental disorders.	0.728	0.627	
	7	Brain malfunctioning may cause the development of mental disorders.	0.693	0.662	
	15	One of the symptoms of depression is the loss of interest or pleasure in most things.	0.668	0.587	
	8	Highly stressful situations may cause mental disorders.	0.621	0.596	
	16	Alcohol use may cause mental disorders.	0.613	0.567	
	14	The symptoms' length is one of the important aspects to determine whether a person has, or has not a mental disorder.	0.604	0.562	
	3	A person with depression feels very miserable.	0.573	0.601	
	17	A person with anxiety disorder avoids situations that may cause her/his distress.	0.551	0.557	
	18	Anorexia nervosa is a type of eating disorder that can lead to death.	0.491	0.491	
	13	A person with an anxiety disorder may panic in situations that she/he fears.	0.487	0.625	
	4	In bulimia nervosa, to compensate for overeating and to prevent weight gain, the person is forced to vomit or exercise vigorously, or use laxatives inappropriately.	0.443	0.493	
First aid skills and help-seeking behavior	21	If a friend of mine developed a mental disorder, I would encourage her/him to look for a psychologist.	0.774	0.621	1.49
	20	If I had a mental disorder, I would seek professional help (psychologist and/or psychiatrist).	0.771	0.637	
	19	If a friend of mine developed a mental disorder, I would encourage her/him to go to a doctor.	0.687	0.463	
	12	If I had a mental disorder, I would seek my family's help.	0.588	0.627	
	26	If a friend of mine developed a mental disorder, I would offer her/his support.	0.567	0.626	
	22	If a friend of mine developed a mental disorder, I would talk to the form teacher or another teacher.	0.515	0.604	
	24	If a friend of mine developed a mental disorder, I would talk to her/parents.	0.489	0.604	
Self-help strategies	9	Good sleep helps to improve mental health.	0.629	0.396	1.29
	2	Doing something enjoyable helps to improve mental health.	0.599	0.441	
	11	Having a balanced diet helps to improve mental health.	0.569	0.683	
	10	Physical exercise helps to improve mental health.	0.564	0.634	
	1	Talking over problems with someone helps to improve mental health.	0.451	0.337	

**Table 3:** The indicators of fitness of the factor analysis of the AMHLQ.

Structure fitness indicators	*χ* ^2^	*df*	*χ* ^2^/*df*	GFI	AGFI	IFI	TLI	CFI	NFI	RMSEA
Four-dimensional structure	1343.281	455	2.963	0.91	0.90	0.90	0.90	0.91	0.90	0.07

GFI: Goodness of fit index; AGFI: Adjusted goodness of fit index; IFI: Incremental fit index; TLI: Tucker-Lewis fit index; CFI: Comparative fit index; NFI: Normal fit index; RMSEA: Root mean square error of approximation.

**Table 4:** Descriptive characteristics of AMHLQ and SDQ.

Descriptive indicators	Mean	Standard deviation	Minimum value	Maximum value
Knowledge of mental health problems	21.76	9.09	10	50
Erroneous beliefs/stereotypes	22.97	9.11	11	49
First aid skills and help-seeking behavior	17.14	7.11	7	35
Self-help strategies	10.71	4.33	5	24
Total mental health literacy	72.59	25.26	33	138
Strengths and difficulties questionnaire	28.31	4.01	18	42

**Table 5:** Concurrent validity of the Persian version of the AMHLQ.

	Total mental health literacy	Knowledge of mental health problems	Erroneous beliefs/stereotypes	First aid skills and help-seeking behavior	Self-help strategies
Strengths and difficulties questionnaire	-0.174∗∗	-0.145∗	-0.150∗	-0.155∗∗	-0.139∗

*p* < 0.0∗.*p* < 0.05∗∗.

**Table 6:** The reliability coefficients of the dimensions of the AMHLQ.

	Cronbach's alpha	Split-half
Total mental health literacy	0.94	0.87
Knowledge of mental health problems	0.89	0.83
Erroneous beliefs/stereotypes	0.89	0.83
First aid skills and help-seeking behavior	0.86	0.79
Self-help strategies	0.74	0.70

## Data Availability

The data used to support the findings of this study are available from the corresponding author upon request.
